The article "MRI View of Rehabilitation Methods to Relieve Anterior Cruciate Ligament Injury in Dancers" was retracted in 2023. Reasons: signs of a paper mill; compromised peer review; unreliable results or conclusions.

# MRI View of Rehabilitation Methods to Relieve Anterior Cruciate Ligament Injury in Dancers

**DOI:** 10.1155/2022/1544440

**Published:** 2022-09-14

**Authors:** Pin Yang

**Affiliations:** Hunan Institute of Engineering, Xiangtan, Hunan 411104, China

## Abstract

In order to solve the problem of the difference in the diagnostic effect of different sequences of magnetic resonance imaging (MRI) examinations for anterior and posterior cruciate ligament injuries, the author proposes an MRI rehabilitation method to relieve anterior cruciate ligament injury in dancers. This method retrospectively analyzed the clinical data of 60 patients with knee anterior and posterior cruciate ligament injuries in our hospital, and all patients were diagnosed with knee anterior and posterior cruciate ligament injuries. All patients underwent MRI 3D sequence and 2D sequence examination successively to compare anatomical measurements. This study aimed at comparing the measurements of the posterior cruciate ligament (PCL) and anterior cruciate ligament (ACL) between the two examination sequences; comparing the diagnosis; comparing the grading and judgment of the anterior and posterior cruciate ligament injuries of the knee joint between the two inspection sequences; and comparing the diagnostic coincidence rates of the two examination sequences in the complete tear of the anterior and posterior cruciate ligaments of the knee. Experimental results show that, in terms of PCL and ACL, the angle, thickness, and length of two-dimensional MRI examination were significantly different from those of MRI examination and anatomical measurement (*P* < 0.05); for PCL and ACL, the angle, thickness, and length of 3D MRI were not significantly different from anatomical measurements (*P* > 0.05). The diagnostic accuracy of 2D MRI was 83.33%, which was lower than 95.00% of 3D MRI (*P* < 0.05). There was no significant difference in the grading of anterior and posterior cruciate ligament injuries between the two examination sequences (*P* > 0.05). The diagnostic coincidence rates of 3D MRI and 2D MRI for complete tear of the anterior and posterior cruciate ligaments were 95.55% and 80.00%, respectively (*P* < 0.05). In conclusion, three-dimensional MRI examination can obtain higher diagnostic value for patients with knee joint anterior and posterior cruciate ligament injury.

## 1. Introduction

Sports dance is an emerging sport with strong technical and artistic qualities; it integrates art, sports, music, and dance, and it is called a model of the combination of “health” and “beauty” [1]. While the male and female players showed vigorous sports movements, it is also necessary to show the attractive artistic beauty of dance movements. The causes of sports injuries in sports dance are closely related to the lack of common knowledge of sports injuries among coaches and students [2]. Due to the lack of basic knowledge of sports injuries and the lack of knowledge of various preventive measures, the cause of the injury cannot be properly analyzed and lessons learned in the event of an injury, resulting in the frequent occurrence of the same injury.

The article "MRI View of Rehabilitation Methods to Relieve Anterior Cruciate Ligament Injury in Dancers" was retracted in 2023. Reasons: signs of a paper mill; compromised peer review; unreliable results or conclusions.

In order to achieve outstanding competition results in sports dance, first of all, in order to ensure the health of the body, it is necessary to have sufficient muscle strength, such as explosive power, balance, coordination, and good quality and state [3]. At the same time, it can avoid the occurrence of sports injury or reduce the degree of injury. In addition, for different types of sports dance, we should pay attention to strengthening the exercise of weak parts and weak links, improve local functions, and meet special requirements. Dance sports is a contest of strength and beauty. In dancing, athletes make good use of loose knee force, strong leg strength and waist, and abdominal strength to make some difficult technical movements [4]. However, the artistry of the project requires the athletes to have the beauty of muscular lines, upright posture, and the perfect combination of strength and beauty. Therefore, correct grasp of the priority order of muscle strength, coordination in the relationship between strengths, improvement in the processing ability of muscles, improvement in the internal coordination ability of muscles, and exercises that avoid muscle bulk and weight gain are especially important [5].

Sports injury (Figure 1) is a common situation for sports dancers in training or competition; it is due to the poor quality of the athletes or mistakes in technical movements; excessive exercise in teaching, sports training, and competition; insufficient preparation for warm-up activities; the venue, equipment, and clothing not meeting the requirements; and factors such as improper organization and management of competition events [6]. Injuries that occur during training have not been adequately rested and properly treated, and you have to continue training with the injury or without waiting for the injury to heal, over time, which will cause the injury to worsen, and this will directly affect the improvement of the level of sports dancers [7]. The injury problem of sports dancers should arouse the great attention of sports dance teachers and sports dancers, improve their awareness of injury prevention, and avoid the occurrence of sports injuries [8]. For this highly technical and artistic combination of sports and dance, sports injuries often trouble and restrict the normal performance of players [9]. Therefore, it is very important to study the sports injury of sports dance.

The article "MRI View of Rehabilitation Methods to Relieve Anterior Cruciate Ligament Injury in Dancers" was retracted in 2023. Reasons: signs of a paper mill; compromised peer review; unreliable results or conclusions.

## 2. Literature Review

The cruciate ligament of the knee joint is also called the cruciate ligament clinically; it is mainly located in the latter part of the center of the knee joint, it has high strength and is covered by the synovial membrane, and it is mainly divided into anterior cruciate ligament and posterior cruciate ligament [10]. The two ligaments work together to limit excessive knee movement. However, knee cruciate ligament injuries are more common after a sports injury or injury from other factors. Due to the low self-healing ability of the cruciate ligament of the knee joint, after the injury, if it is not diagnosed in time and effective measures are taken to intervene, it is very easy to develop into a complete tear, which will adversely affect the stability of the joint, called secondary traumatic osteoarthropathy [11]. MRI is a commonly used imaging examination method in clinical practice; it has played a good role in the diagnosis of various diseases, it can achieve parametric and multidirectional imaging, and it has strong advantages in displaying articular cartilage and intra-articular structures. However, there are few studies on the difference in the effect of different examination sequences in the diagnosis of knee cruciate ligament injury, which limits the rational selection of clinical examination sequences to a certain extent. The three-dimensional fast spin echo sequence has the characteristics of high signal-to-noise ratio and high spatial resolution, which can realize thin-slice and no interval scanning and then clearly display the complex joint anatomy, which can play an important reference value in judging soft tissue damage.

Anterior cruciate ligament injury is one of the common diseases of the knee joint, which can lead to complications such as knee joint rotation imbalance, osteoarthritis, and cartilage degeneration; due to the early symptoms of joint swelling and pain in patients after injury, imaging diagnosis has caused certain difficulties. MRI is currently the main imaging method for diagnosing anterior cruciate ligament injury; however, there are still great limitations in diagnosing based on MRI signal intensity changes, resulting in low accuracy and specificity in the diagnosis of partial anterior cruciate ligament tear, which seriously affects the anterior cruciate ligament injury and the early diagnosis and treatment of cruciate ligament injury. Diffusion tensor imaging (DTI), as a quantitative diagnostic imaging technique, has so far been mainly used in the clinical diagnosis of central nervous system lesions; however, with the gradual popularization of DTI technology, there have been reports locally and abroad that it has been applied to other soft tissue lesions other than the central nervous system, along with the use of MRI and DTI to study normal anterior cruciate ligament and anterior cruciate ligament injury reconstruction. Moreover, there are few DTI studies on the grading of cruciate ligament injury; the application of DTI-based tractography (DTT) to evaluate the diagnostic effect of different grades of anterior cruciate ligament injury has not been seen [12]. In this study, DTI and DTT techniques were used to observe the fractional anisotropy (FA) value and apparent diffusion coefficient (ADC) value of the anisotropy fraction (FA) and apparent diffusion coefficient (ADC) of the injured anterior cruciate ligament and the corresponding parts of the normal group and with different degrees of injury, and its correlation with the degree of injury, in order to compare the diagnostic value of DTT in grading the degree of anterior cruciate ligament injury.

The article "MRI View of Rehabilitation Methods to Relieve Anterior Cruciate Ligament Injury in Dancers" was retracted in 2023. Reasons: signs of a paper mill; compromised peer review; unreliable results or conclusions.

The author conducted a retrospective analysis of the clinical data of patients with cruciate ligament injury of the knee joint who underwent MRI examination in our hospital and were clinically diagnosed; the research content is described as follows [13].

## 3. Methods

### 3.1. Research Objects and Methods

#### 3.1.1. Research Objects

The clinical data of 60 patients with knee anterior and posterior cruciate ligament injuries were retrospectively analyzed in a hospital, the inspection time was between January 2020 and January 2021, and all patients were diagnosed with anterior and posterior knee injuries such as cruciate ligament injury. Among the 60 patients, 28 were female and 32 were male; the age ranged from 25 to 45 years, and the average age was 32.71 ± 4.15 years. Injury factors were 24 cases of traffic accidents, 15 cases of falling from heights, 13 cases of heavy objects smashing, and 8 cases of other reasons; There were 45 complete tears and 15 partial tears [14].

The inclusion criteria were as follows: (i) clinical manifestations and surgical results were all diagnosed as anterior and posterior cruciate ligament injury; (ii) the clinical data were complete; (iii) the compliance was good, and the patients were able to cooperate with the examination; (iv) the affected knee joint had swelling, pain, and movement disorders; and for performance, (v) drawer test results were positive.

The exclusion criteria were as follows: (i) patients who have undergone knee surgery; (ii) women who are pregnant or breastfeeding; (iii) those who have a history of severe fractures; (iv) those who have a history of rheumatoid arthritis; (v) those who have tumor diseases; (vi) those who have congenital bone deformities; and (vii) patients with heart, liver, kidney, and lung organic function damage.

The article "MRI View of Rehabilitation Methods to Relieve Anterior Cruciate Ligament Injury in Dancers" was retracted in 2023. Reasons: signs of a paper mill; compromised peer review; unreliable results or conclusions.

#### 3.1.2. Research Methods

All patients were examined using the MAGNETOM Skyra 3.0 T magnetic resonance imaging system, using a special coil for the knee joint. The patients were assisted in a supine position and instructed to externally rotate the knee by 15° and maintain this angle during the examination. The 2D MRI scan parameters were as follows: (i) For the horizontal axis, the repetition time is 2000 ms, the recovery time is 38 ms, the matrix is 300 × 230, the field of view is 150 mm × 150 mm, the layer spacing is 0.5 mm, the layer thickness is 2.8 mm, the scanning time is 160 s, and the number of excitations is 2. (ii) For the sagittal plane, the repetition time is 2900 ms, the recovery time is 30 ms, the matrix is 240 × 240, the field of view is 155 mm × 155 mm, the slice interval is 0.41 mm, the slice thickness is 2.4 mm, the scanning time is 150 s, and the number of excitations is 2 times. (iii) For the coronal plane, the repetition time is 2600 ms, the recovery time is 30 ms, the matrix is 300 × 230, the field of view is 155 mm × 155 mm, the layer spacing is 0.41 mm, the layer thickness is 2.4 mm, the scanning time is 160 s, and the number of excitations is 2 times. The 3D MRI scanning parameters were as follows: for the sagittal plane, the repetition time is 1100 ms, the recovery time is 38 ms, the matrix is 300 × 230, the field of view is 150 mm × 150 mm, the slice spacing is 0 mm, the slice thickness is 0.5 mm, the scanning time is 320 ms, and the number of excitations is 1 time [15]. After three-dimensional MRI scans, all images were reconstructed in all planes, with a slice thickness of 1.5 mm and a slice interval of 0 mm. The operation was performed by 2 radiologists with rich clinical experience, and the images were read together to judge the knee joint injury situation and degree; when there was disagreement, a unified conclusion could be reached after discussion.

### 3.2. Research and Analysis

#### 3.2.1. Observation Items

The posterior cruciate ligament (PCL) and anterior cruciate ligament (ACL) measurements were compared between the two examination sequences. The diagnosis of the two examination sequences were compared, as well as the grading and judgment of the anterior and posterior cruciate ligament injuries of the knee joint between the two inspection sequences. The contour and direction of the anterior and posterior cruciate ligaments of the knee joint were normal, and no abnormal signal was observed, which belonged to grade 0. Focal or diffuse swelling of the anterior and posterior cruciate ligaments of the knee joint as well as a high signal can be observed, the ligament continuity is acceptable, and the contour is clear and no notch is classified as grade 1. Incomplete rupture of the anterior and posterior cruciate ligaments of the knee joint as well as a thickening of the ligament can be observed, local notch may be present, the contour at the center of the injured area is incomplete, the ligament is interrupted, and the continuity is poor, but there are still some ligament connections belonging to grade 2. The anterior and posterior cruciate ligaments of the knee joint were completely ruptured, and the rupture site was incised or displaced, contracture at the ligament origin and insertion point was observed, and different degrees of dissolution and absorption at the rupture site belonged to grade 3. The diagnostic coincidence rates of the two examination sequences in the complete tear of the anterior and posterior cruciate ligaments of the knee were compared [16].

The article "MRI View of Rehabilitation Methods to Relieve Anterior Cruciate Ligament Injury in Dancers" was retracted in 2023. Reasons: signs of a paper mill; compromised peer review; unreliable results or conclusions.

#### 3.2.2. Athletes' Assessment of Injury Risk from Sports Injuries

It is shown in Table 1 that among the physical factors of sports dance professional athletes, injury history, physical fatigue, poor physical condition, and poor flexibility are the moderate risk factors for injury. The movement range of sports dance is large and flexible, and most of the sports dance movements are in contradiction with the anatomical structure of the human body; for example, most movements require a large range of motion and high flexibility of the hip joint, amplitude, and flexibility, directly affecting the quality of dance postures and technical movements. Moreover, the anatomical structure of the hip joint is characterized by good joint stability and poor flexibility; for example, the athlete's flexibility quality is poor, and when forcibly performing large-scale and high-speed hip joint movements that exceed the body's tolerance limit, it is easy to cause corresponding damage to the site [17]. The above four factors remind coaches and athletes that they should pay enough attention. Poor physical coordination, strength, and endurance are low-risk factors and are acceptable risks, but they cannot be ignored in normal training.

From Table 2, it can be seen that among the risk factors of injury caused by technical factors of sports dance professional athletes, incorrect technical essentials and improper self-prevention measures for injury are medium risk factors, and improper cooperation between dance partners and dance style are low. The risk factor is the incorrect technical essentials which refer to the damage to the body tissue caused by the athlete's technical shortcomings and mistakes, violating the characteristics of the human body structure and the laws of activity of various organ systems, as well as the mechanical principles during exercise.

The article "MRI View of Rehabilitation Methods to Relieve Anterior Cruciate Ligament Injury in Dancers" was retracted in 2023. Reasons: signs of a paper mill; compromised peer review; unreliable results or conclusions.

From Table 3, it can be seen that among the psychological factors of sports dance professional athletes, inattention and excessive mental stress are medium risk factors for injury, while depression and high excitement during training or competition are low risk factors. The research of domestic and foreign scholars shows that psychological factors are not only related to the performance of sports performance but also directly related to the pathogenesis of sports injuries.

From Table 4, it can be seen that among the risk of injury caused by other factors of professional dance athletes, accidents and emergencies are ranked first, followed by irregular life and rest, collisions during competitions, and referee factors; the above four factors are all low-risk factors, which are acceptable risks [18]. Accidents and emergencies are unforeseeable and mainly reflect the ability of athletes to respond to stress; for example, in research on the relationship between the stress level and sports injuries of sports students, high stress levels are one of the important causes of sports injuries. Athletes with high levels of stress are more easily affected by the external environment, such as obstacles to marriage and love, the death of relatives and friends, and emergencies on the training ground or on the field, all of which can affect the emotional state of athletes, thus affecting the physiological state and attention, so that sports injuries are prone to occur, and irregular life and rest can easily lead to the athletes' decline in function and easy fatigue, thereby increasing the risk of injury.

Based on the assessment results of the injury risk of professional sports dance athletes in the above four dimensions, we can see the main characteristics of the injury risk of sports dance athletes; the most important injury risks of athletes during training or competition are as follows: injury training or competition, injury history, physical fatigue, partial overload, incorrect technical essentials, poor physical condition, inattention, etc. (Figure 2). This is basically consistent with the results of the open-ended questionnaire Pareto analysis. Athletes should take different preventive measures when dealing with different injury risks [19]. Coaches and athletes can generally take two types of measures when preventing injuries: risk avoidance and risk reduction. Among all the factors investigated, coaches and athletes generally believe that training or competition with injuries is the most likely to lead to the occurrence of injuries; therefore, for such risk factors, it is necessary to consider giving up training or competitions, or change the original training program to avoid risks. Excessive partial load or excessive exercise load on the body can easily lead to physical fatigue, resulting in decreased function and injury; therefore, coaches should scientifically arrange training plans to control exercise load, and especially to avoid single repetition of the same part of the training to reduce local burden to reduce the risk of injury [20]. Technical errors or mistakes are also the main cause of injury, so athletes should standardize their movements in their usual training and strengthen the learning of correct technical essentials, thereby reducing the risk of injury. Among the psychological factors, factors such as inattention and excessive mental tension may also lead to the occurrence of injuries such as technical deformation or errors in athletes during training and competition; for such factors, prevention and response should start from normal, strengthening the training of psychological adjustment ability to reduce the risk.

The article "MRI View of Rehabilitation Methods to Relieve Anterior Cruciate Ligament Injury in Dancers" was retracted in 2023. Reasons: signs of a paper mill; compromised peer review; unreliable results or conclusions.

#### 3.2.3. Data Processing

In this study, the data were calculated using SPSS22.0 software, and the measurement data were expressed in the form of ($\bar{x}\pm s$), the *t* test was implemented, and the *F* value test was implemented for comparison between multiple groups. The enumeration data is expressed in the form of percentage, and the *X*^2^ test is implemented; when the test result shows *P* < 0.05, it indicates that the data has research value [21].

## 4. Results and Discussion

In terms of PCL and ACL, the angle, thickness, and length of two-dimensional MRI examination were significantly different from those of MRI examination and anatomical measurement (*P* < 0.05) [22, 23]. In terms of PCL and ACL, the angle, thickness, and length of 3D MRI were not significantly different from the anatomical measurements (*P* > 0.05). See Tables 5 and 6.

## 5. Conclusion

The author proposes the MRI view of rehabilitation methods to relieve ACL injury in dancers. The main risks of injury caused by sports dancers are as follows: injury training or competition, injury history, physical fatigue, partial overload, incorrect technical essentials, poor physical condition, inability to concentrate, etc. Athletes can take different preventive measures when dealing with different risks of injury; generally, two types of measures can be taken: risk avoidance and risk reduction. Among them, risk reduction is the most widely used preventive coping strategy for athletes.

The article "MRI View of Rehabilitation Methods to Relieve Anterior Cruciate Ligament Injury in Dancers" was retracted in 2023. Reasons: signs of a paper mill; compromised peer review; unreliable results or conclusions.

## Figures and Tables

**Figure 1:** Ligament injury.

**Figure 2:** The main risks of injury caused by professional dance sports athletes.

**Table 1:** Risk assessment results of physical factors for sports dance professional athletes.

Physiological factors	Amount of risk (Rv)	Risk level	Risk warning signs	Sort
Poor health (such as illness)	43.25 ± 15.42	Medium risk	Yellow	3
Injury history	62.25 ± 31.74	Medium risk	Yellow	1
Physical fatigue	49.63 ± 31.76	Medium risk	Yellow	2
Poor strength	29.25 ± 16.91		Green	6
Poor endurance	25.50 ± 17.72	Low risk	Green	7
Poor flexibility	40.75 ± 17.95	Medium risk	Yellow	4
Poor coordination	37.88 ± 19.67	Low risk	Green	5

**Table 2:** Risk assessment results of technical factors for sports dance professional athletes.

Physiological factors	Amount of risk (Rv)	Risk level	Risk warning signs	Sort
Incorrect technical essentials	45.25 ± 9.79	Medium risk	Yellow	1
Dance style	25.63 ± 12.05	Low risk	Green	4
Improper cooperation between dance partners	30.38 ± 4.84	Low risk	Green	3
Improper self-prevention measures	41.75 ± 11.88	Medium risk	Yellow	2

**Table 3:** Risk assessment results of psychological factors for sports dance professional athletes.

Physiological factors	Amount of risk (Rv)	Risk level	Risk warning signs	Sort
Feeling down during training or competition	37.00 ± 19.09	Low risk	Green	3
Excessive excitement during training or competition	32.75 ± 9.19	Low risk	Green	4
Inattention	42.75 ± 11.56	Medium risk	Yellow	1
Nervousness	40.13 ± 13.25	Medium risk	Yellow	2

**Table 4:** Risk assessment results of other factors for sports dance professional athletes.

Physiological factors	Amount of risk (Rv)	Risk level	Risk warning signs	Sort
Referee factor	11.88 ± 5.19	Low risk	Green	4
Irregular life	35.13 ± 16.14	Low risk	Green	2
Collision during game	29.50 ± 10.93	Low risk	Green	3
Accident, accident	36.00 ± 17.63	Low risk	Green	1

**Table 5:** PCL measurement values of two groups of inspection sequences.

Check the sequence	Number of cases	Angle (°)	Thickness (cm)	Length (cm)
2D MRI	60	119.62 6.51	0.71 0.07	3.82 0.31
3D MRI	60	115.70 5.03	0.53 0.04	3.71 0.19
Anatomical measurements	60	115.53 5.12	0.52 0.03	3.70 0.24
*F*	—	10.260	278.110	4.200
*P*	—	<0.05	<0.05	<0.05
*X* ^2^_1_/*P*_1_	—	3.825/<0.05	19325/<005	2.371/<0.05
*X* ^2^_2_/*P*_2_	—	0.235/>0.05	1.560/>0.05	0.308/>0.05
*X* ^2^_3_/*P*_3_	—	3.691/<0.05	17.294/<0.05	2.343/<0.05

**Table 6:** ACL measurement values of the two groups of examination sequences.

Check the sequence	Number of cases	Angle (°)	Thickness (cm)	Length (cm)
2D MRI	60	37.40 4.18	0.73 0.05	3.22 0.11
3D MRI	60	39.35 4.98	0.63 0.02	3.57 0.16
Anatomical measurements	60	39.38 4.93	0.62 0.04	3.62 0.25
*F*	—	3.480	148.000	85.330
*P*	—	<0.05	<0.05	<0.05
*X* ^2^_1_/*P*_1_	—	2.373/<0.05	13307/<005	11.344/<0.05
*X* ^2^_2_/*P*_2_	—	0.049/>0.05	2.000/>0.05	2.1 19/>005
*X* ^2^_3_/*P*_3_	—	2.323/<0.05	14.384/<0.05	13.963/<005

The article "MRI View of Rehabilitation Methods to Relieve Anterior Cruciate Ligament Injury in Dancers" was retracted in 2023. Reasons: signs of a paper mill; compromised peer review; unreliable results or conclusions.

## Data Availability

The data used to support the findings of this study are available from the corresponding author upon request.
